This article has been retracted.

# Circular RNA circHIPK3 Promotes Cell Metastasis through miR-637/STAT3 Axis in Osteosarcoma

**DOI:** 10.1155/2020/2727060

**Published:** 2020-07-24

**Authors:** Zhongyue Huang, Chunyan Yuan, Huijie Gu, Xiangyang Cheng, Kaifeng Zhou, Jun Xu, Xiaofan Yin, Jiangni Xia

**Affiliations:** ^1^Department of Orthopaedics, Minhang Hospital, Fudan University, 170 Xin-Song Road, Shanghai 201199, China; ^2^Department of Pathology, Minhang Hospital, Fudan University, 170 Xin-Song Road, Shanghai 201199, China

## Abstract

Recent studies have suggested that circular RNAs play an important role in the progression of various cancers. However, few studies have revealed the great value of circRNAs in the diagnosis and prognosis prediction of osteosarcoma (OS). In this study, we performed experiments with the human OS cell lines and the results showed that the expression of circHIPK3 in OS cell lines was significantly upregulated compared to that in the normal cell line. In addition, the results showed that circHIPK3 could promote the migration, invasion, and growth of OS cells. Furthermore, miR-637 was identified as a target of circHIPK3, while STAT3 was targeted by miR-637. circHIPK3 could promote STAT3 expression via interacting with miR-637 in OS cells. In conclusion, our research uncovered an important role of the circHIPK3/miR-637/STAT3 pathway in the migration and invasion of OS cells and suggested that circHIPK3 may be a prognostic marker and a promising therapeutic target for OS.

## 1. Background

Osteosarcoma (OS) is a primary malignancy that develops in the long bones of the extremities [1]. The incidence of OS worldwide is approximately one to three cases per million people per year [2]. OS is characterized by a difficult etiology, high-frequency local invasion, and rapid metastatic potential [3]. Despite advances in treatment technology and medical development, the treatment of osteosarcoma remains one of the challenges facing doctors [4]. Current treatment strategies have failed to make more progress in improving patient survival and quality of life. Therefore, more advanced protocols and drugs are still needed [5].

With the development of technology and further research, various small molecules in cells have been found to be able to regulate cell activities [6, 7]. Among them, circRNA is a kind of RNA without coding potential that has been widely reported to regulate cell growth, metabolism, and metastasis [8, 9] and could be implicated in RNA or protein sponging to modulate gene expression [10]. For example, circRNA HRCR serves as a miR-223 sponge to suppress its activity, thereby repressing miR-223's target expression and ultimately inhibiting cardiac hypertrophy and heart failure [11]. Circ-abcb10 was found to have a spongy effect on miR-1271 in breast cancer cells, promoting cell proliferation and inhibiting cell apoptosis [8]. Circ_101222 in blood cells can be used to predict early preeclampsia [9]. circRNA_102171 overexpression promotes PTC progression through activating the Wnt/*β*-catenin pathway in a CTNNBIP1-dependent way [12].

circHIPK3 consists of two targeting sites of miR-558, and the binding between circHIPK3 and miR-558 could significantly inhibit the expression of heparinase, thereby reducing the invasion, migration, and angiogenesis of cancer cells [13]. Meanwhile, circHIPK3 can decrease miR-7 in colorectal cancer cells, thus promoting the growth, migration, and invasion of colorectal cancer cells [14]. It has also been shown that silencing circHIPK3 suppresses the growth of liver cancer cells while ectopic overexpression of circHIPK3 can promote the growth of gallbladder cancer cells [15, 16]. However, the roles of circHIPK3 in OS remained unclear.

In vitro functional assay showed that circHIPK3 can promote the proliferation of osteosarcoma cells and enhance cell migration and invasion. We found that circHIPK3 could sponge on miR-637, thus significantly reducing the effect of miR-637 on its downstream gene STAT3, thus promoting the growth and spread of cancer cells.

## 2. Materials and Methods

### 2.1. Patient Samples

Ten patients with OS were included in our study with written informed consent. Both the matched noncancerous tissues and OS tissues were obtained from each patient. The project was approved by the research ethics committee of Minhang Hospital, Fudan University.

### 2.2. Cell Culture and Transfection

U2OS and SW1353 cells were from ATCC and maintained in RPMI-1640 medium with 10% FBS. Cells were transfected with circHIPK3 siRNA (si-circHIPK3) (GenePharma, Suzhou, China) and control siRNA (si-NC) using Lipofectamine 2000 (Thermo Fisher Scientific) [17].

### 2.3. qRT-PCR Analysis

Total RNA was isolated from OS samples using TRIzol reagent. Total RNA was reverse transcribed to cDNA, and then, qPCR was conducted by using a SYBR Green PCR Kit (Takara, Otsu, Japan). All primer sequences were designed and synthesized by GenePharma (Shanghai, China). GAPDH was chosen as the reference gene for circRNA and mRNA. Gene expression was calculated with the 2^−*ΔΔ*Ct^ method.

### 2.4. Cell Invasion and Cell Migration

A Transwell plate coated with Matrigel or without Matrigel was used for cell invasion assays or migration assays. The cells were precultured in a serum-free medium for 6 hours and then resuspended seeded to the upper chamber of the Transwell in a medium containing 1% FBS, and the medium containing 20% FBS in the lower chamber was used as the chemoattractant. After incubation for 48 hours, Matrigel and the cells in the upper chamber were removed and the cells on the lower surface were fixed and stained with DAPI (Solarbio, Beijing, China). The cell number was counted in 5 random microscopic fields (×200).

### 2.5. CCK-8 Assay

Cells were seeded in 96-well plates and CCK-8 (10 *μ*l/well) was added; the absorbance OD 450 of each well was measured with a microplate reader after incubation for 2 hours [18].

### 2.6. Dual-Luciferase Reporter Assay

The miR-637 target sequence in circHIPK3 or STAT3 was amplified and inserted into the luciferase vector. 293T cells were transfected with Wt/Mut-circHIPK3 or Wt/Mut-STAT3 and miR-637 mimics or control miRNA (miR-NC) using Lipofectamine 2000 (Invitrogen) [19]. The luciferase activities were measured through the Dual-Luciferase Assay System (Promega).

### 2.7. Statistical Analysis

The analysis of experimental data was calculated with SPSS 19.0 statistical software. The comparison between the two groups was calculated using Student's *t*-test or the one-way analysis of variance (ANOVA) method. We considered *p* < 0.05 was statistically significant [20].

## 3. Results

### 3.1. circHIPK3 Was Upregulated in OS Tissues and Cells

Through qPCR assay, we found that circHIPK3 was significantly upregulated in OS tissues and cell lines compared to that in control tissues and cells (Figures 1(a) and 1(b)) (*p* < 0.001).

### 3.2. Knockdown of circHIPK3 Inhibited OS Cell Proliferation

To investigate circHIPK3's role in osteosarcoma, we examine U2OS and SW1353 cell proliferation rate after circHIPK3 knockdown using CCK-8 assay. The result showed that the cell growth rate of U2OS and SW1353 cells was significantly suppressed after circHIPK3 knockdown compared to the negative control group in series time points (Figures 2(a) and 2(b)), demonstrating that circHIPK3 could promote OS cell proliferation. The knockdown efficiency is shown in Figure 1(c).

### 3.3. Knockdown of circHIPK3 Inhibited OS Cell Migration and Invasion

We further performed a Transwell assay to investigate the functional roles of the circHIPK3 role in OS progression. The result showed that the silencing of circHIPK3 greatly inhibited U2OS and SW1353 cell migration and invasion compared to control groups (Figures 2(c)–2(f)).

### 3.4. circHIPK3 Promoted STAT3 Expression by Reducing miR-637 in OS through Sponging

Using localization analysis, circHIPK3 is reported to be mainly located in the cytoplasm (Figures 3(a) and 3(b)). To explore the mechanisms, we next analyzed the downstream targets of circHIPK3 through bioinformatics analysis and found circHIPK3 may bind to miR-637. Luciferase reporter assay demonstrated the luciferase activity was significantly reduced in 293T cells after the cotransfection of miR-637 mimic with Wt-circHIPK3. We also showed no significant difference after cells cotransfected with miR-637 mimic and Mut-circHIPK3 (Figure 3(c)). Moreover, knockdown of circHIPK3 induced a significant increase of miR-637 in both SW1353 and U2OS cells (Figure 3(d)). Interestingly, we found miR-637 could suppress circHIPK3 levels in OS cells (Figure 3(e)).

Previous studies suggested that STAT3 is one potential target site of miR-637. To verify the interaction between miR-637 and STAT3, we cloned the 3′UTR of STAT3 or mutant sequences into the pmirGLO vector and then cotransfected into 293T with miR-637 mimic or negative controls. Luciferase activity was significantly lower in cells cotransfected with miR-637 mimic and Wt-STAT3 than that in cells with negative controls (Figure 4(a)). Besides, miR-637 significantly decreased STAT3 expression in OS cells (Figure 4(b)). To further explore the relationship among circHIPK3, miR-637, and STAT3, OS cells were cotransfected with si-circHIPK3 and si-miR-637. qRT-PCR assays showed that si-circHIPK3 decreased STAT3 expression in OS cells, while si-miR-637 weakened the effects (Figures 4(c) and 4(d)). The above results indicated that circHIPK3 may regulate OS progression through the circHIPK3/miR-637/STAT3 axis.

## 4. Discussion

circHIPK3 is a circRNA produced by direct reverse splicing of the coding sequence of the HIPK3 gene [21]. circHIPK3 has an intracellular half-life of more than 24 hours, indicating its resistance to nucleic acid exonuclease [22]. Studies have reported that in seven types of cancers including bladder epithelial carcinoma [13], prostate cancer [23], colorectal cancer [14], and six types of normal tissues, circHIPK3 was highly expressed. It was found that circHIPK3 contained more than one binding site of multiple miRNAs, which could inhibit the activity of miRNA [24]. Previous reports have shown circHIPK3 is abundant in multiple cancers and can enhance the growth of cancer cells [25–27]. For example, in oral squamous cell carcinoma, downregulation of the circHIPK3 gene can reduce the adsorption of miR-124, which can normally regulate the downstream target gene and suppress cancer cell growth [28]. circHIPK3 is an inhibitor of miR-4288 in nasopharyngeal carcinoma cells, which can inhibit the expression level of the latter, thereby enhancing the expression of ELF3 and promoting the malignant progress of nasopharyngeal carcinoma cells [26]. In addition, circHIPK3 also plays a role in senile cataracts. The silencing of circHIPK3 in human lens epithelial cells increased the expression of miR-193a, significantly accelerated the apoptosis of human lens epithelial cells under oxidative stress, and inhibited cell proliferation [25]. circHIPK3 is also highly expressed in human lung tissues, inhibiting miR-338-3p activity through serving as an endogenous miR-338-3p sponge, improving the fibroblast-to-myofibroblast transition, and inhibiting the proliferation of fibroblasts [27]. However, circHIPK3 shows different effects in some cells. According to studies in bladder cancer, circHIPK3 is significantly downregulated in bladder cancer, which leads to the adsorption of miR-558 that is significantly weakened, leading to a decreased targeting effect of miR-558 on the heparinase gene, thereby promoting bladder cancer progression. In contrast, the forced overexpression of circHIPK3 reverses these regulatory processes and inhibits the growth and development of bladder cancer cells [13]. In the present study, we found that circHIPK3 was overexpressed in OS tissues and cell lines and acted as an oncogene in OS by promoting cancer cell proliferation, migration, and invasion.

miRNAs are characterized by their small molecular weight, consisting of approximately 22 ribonucleotides [29]. miRNAs mainly play a regulatory role in cells, regulating the translation process by binding to specific sites of mRNA and affecting the expression of related genes [30]. Most circRNAs were found to have sites homologous with miRNAs and can act as sponges to adsorb target miRNAs, thus inhibiting the miRNAs' regulation [31]. Extensive evidence suggests that some circRNAs may act as competitive endogenous RNA (ceRNA) competing with matched miRNAs for binding sites on the latter, thereby affecting the normal functioning of miRNAs. For example, human circRNA can significantly reduce the efficiency of miR-7 binding to its target mRNA by binding to miR-7 as a sponge [32]. More surprisingly, a single circRNA has more than one binding site. For example, studies in a variety of cancer tissues and normal tissues have found that circHIPK3 has up to 18 potential binding sites, which can regulate nine miRNAs from different sources and play the role of sponge [24]. Therefore, circRNAs are complex and powerful, which is also related to their special ring structure. Its stable structure allows it to avoid being rapidly broken down by intracellular degradation mechanisms [33]. Our study found that circHIPK3 can also play a spongy role of miR-637, and the knockdown of circHIPK3 significantly increased the expression of miR-637.

miR-637 can play various roles in cellular processes [34–36]. Exogenous miR-637 can regulate the expression of RING1 in order to intervene to reverse the proliferation of cervical cancer cells mediated by C5orf66-AS1 and inhibit cancer cell growth [36]. miR-637 could regulate c-reactive protein (CRP) in the acute phase. miR-637 competitively binds HuR to CRP mRNA by interacting with CRP 3′UTR to reduce the protein abundance of CRP expression level, which is an important inflammatory marker [35]. In addition, studies have shown that miR-637 inhibits the growth of human mesenchymal stem cells (hMSCs) and induces s-phase arrest. At the same time, miR-637 significantly enhanced adipocyte differentiation in hMSC and inhibited osteoblasts by directly inhibiting Osterix expression, thus playing an important role in maintaining the balance between adipocytes and osteoblasts [34]. Our study found that miR-637 binds to the mRNA of oncogene STAT3 and regulates its expression, respectively, confirmed by double luciferase reporter assay and measured by qRT-PCR. STAT3 has been extensively demonstrated to be activated by structural phosphorylation in v-src transforming cells, which plays a central role in the process of malignant transformation [37]. Therefore, our study suggests that miR-637 can inhibit the growth and development activity of osteosarcoma cells by inhibiting the mRNA activity of STAT3.

In this study, we measured the abnormal increase of circHIPK3 expression in OS samples and cells by qRT-PCR and confirmed that circHIPK3 can promote the growth and metastasis of OS cells (SW1353 and U2OS) in vitro. The above research results. We also proved the mechanism of action of circFAT1 (e2) in osteosarcoma. However, our research still has certain limitations. In follow-up studies, we will conduct animal model experiments and increase the number of clinical samples to further verify that circHIPK3 affects the tumorigenesis and development of osteosarcoma in vivo. Also, we realized there was a lack of comprehensive identification of circRNAs in OS. We plan to collect the clinical samples and apply RNA-sequencing in the future study.

In summary, compared with normal people, we found that circHIPK3 was upregulated in OS. Knocking out circHIPK3 could inhibit the proliferation and metastasis of OS. We further found that circHIPK3 could sponge miR-637, thereby inducing STAT3 expression and promoting OS progression. Also, circHIPK3 played a vital role in the development of osteosarcoma. Our research revealed a novel regulatory pathway in OS, which may provide a new strategy for the diagnosis and treatment of OS.

## Figures and Tables

**Figure 1:** circHIPK3 was upregulated in OS. (a) The expression of circHIPK3 in 10 paired OS tissues was measured by qRT-PCR. (b) Relative expression of circHIPK3 in OS cell lines (U2OS, SW1353) and human osteoblasts (hFOB 1.19). (c) circHIPK3 expression in OS cells transfected with si-circHIPK3 or si-NC. ^∗^*p* < 0.05, ^∗∗^*p* < 0.01, and ^∗∗∗^*p* < 0.001.

**Figure 2:** Knockdown of circHIPK3 decreased OS cell proliferation, invasion, and migration. (a, b) The cell proliferation of U2OS and SW1353 cells transfected with si-circHIPK3 was evaluated by CCK-8. (c–f) Invasion and migration numbers in transfected U2OS and SW1353 cells were evaluated by Transwell assays. ^∗^*p* < 0.05, ^∗∗^*p* < 0.01, and ^∗∗∗^*p* < 0.001.

**Figure 3:** circHIPK3 served as a sponge for miR-637. (a, b) Comparison of the abundance of circHIPK3 in nuclear and cytoplasmic. (c) Luciferase reporter assay showed that miR-637 mimics dramatically reduced luciferase activity of the Wt-circHIPK3 group. (d) miR-637 was enriched by the downregulation of circHIPK3 compared with the negative control. (e) Compared with the control group, miR-637 overexpression downregulated circHIPK3. ^∗^*p* < 0.05 and ^∗∗^*p* < 0.01.

**Figure 4:** STAT3 was a direct target of miR-637. (a) miR-637 mimics significantly reduced the luciferase activity of Wt-STAT3. (b) miR-637 overexpression reduced STAT3 expression levels in U2OS and SW1353 cells. (c, d) miR-637 underexpression rescued the effects of circHIPK3 knockdown on STAT3 expression levels. ^∗^*p* < 0.05.

## Data Availability

The datasets used and/or analyzed during the current study are available from the corresponding author on reasonable request.
